# Ulnar malignant peripheral nerve sheath tumour diagnosis in a mixed-breed dog as a model to study human: histologic, immunohistochemical, and clinicopathologic study

This article has been retracted.

**DOI:** 10.1186/1746-1596-8-86

**Published:** 2013-05-20

**Authors:** Abbas Tavasoly, Javad Javanbakht, Fariba Khaki, Ehsan Hosseini, Alimohammad Bahrami, Mehdi Aghamohammad Hassan, Mohammadmehdi Mirabad

**Affiliations:** 1 Department of Pathology, Faculty of Veterinary Medicines, Tehran University, Tehran, Iran; 2 Paraveterinary Faculty of Ilam, University of Ilam, Ilam, Iran; 3 Department of Clinical Science, Faculty of Veterinary Medicine, Tehran University, Tehran, Iran

**Keywords:** Dog, Pathology, Immunohistochemistry, Tumor, Markers

## Abstract

Canine Malignant Peripheral Nerve Sheath Tumors (MPNSTs) are uncommonly reported in the ulnar, since they are underestimated relative to the more common spindle cell tumours of soft tissue. In dogs, MPNST accounts for 27% of nervous system tumours. In man, MPNST represents 5-10% of all soft tissue sarcomas and is often associated with neurofibromatosis type 1 (NF-1).An 8-year-old, 9 kg, female mixed-breed dog with a subcutaneous mass on the upper right side of the ulnar region was presented to the small animal research and teaching hospital of Tehran University. The dog was anorexic with general weakness. The mass (7 × 4 cm) was removed surgically and processed routinely. Microscopically, the mass was composed of highly cellular areas with a homogeneous population of round or spindle cells, high cellular pleomorphism, high mitotic index and various morphologic patterns. Furthermore, spindle cells arranged in densely or loosely sweeping fascicles, interlacing whorls, or storiform patterns together with wavy cytoplasm, nuclear palisades, and round cells were arranged in sheets or cords with a meshwork of intratumoral nerve fibers. In addition, in this case the presence of neoplastic cells within the blood vessels was observed. Immunohistochemically, tumor was positive for vimentin and S-100 protein. The histopathologic features coupled with the S-100 and vimentin immunoreactivity led to a diagnosis of malignant neurofibroma.

To the best of our knowledge, primary ulnar MPNST has not been reported in animals. This is the first documentation of an ulnar malignant peripheral nerve sheath tumour in a dog.

**Virtual slides:**

The virtual slide(s) for this article can be found here: http://www.diagnosticpathology.diagnomx.eu/vs/1310907815984587

## Background

Canine peripheral nerve sheath tumors (PNSTs) are uncommonly reported, and their clinical behavior has not been well documented [1,2]. These tumors are relatively common in humans but occur infrequently in domestic animals [3]. Based on the morphologic and biologic behavior, PNSTs are divided to benign PNST (BPNST) and malignant PNST (MPNST) forms with several morphologic features [1-3]. MPNST is an aggressive and uncommon neoplasm that develops within peripheral nerve [4].

In human MPNSTs, variable histologic patterns and heterogenous differentiation have been reported [5-7], including epithelioid MPNST [8,9] and MPNST with divergent differentiation such as rhabdomyoblastic (malignant Triton tumor) [10-12] cartilaginous, osseous, angiomatous [13] and glandular forms [14,15], or their complex [16]. Similar representation such as epithelioid type [17], melanotic type [18,19] cartilaginous and osteogenic [20] or glandular epithelial differentiation have been found in MPNSTs in dogs or other animals [3,21].

Histologically, in human MPNSTs, the malignant nature of these tumours were evident upon their microscopic inspection, as they were comprised of an infiltrative and cellular proliferation of atypical, mitotically active spindle cells. Most MPNSTs are high-grade tumours with a high mitotic rate and commonly induce necrosis. The most common histological patterns include a high-grade fibrosarcomatous mass composed of densely packed sheets of plump but relatively uniform spindle or oval cells [4,22-26].

Immunohistochemical studies have contributed to the definition of clear diagnostic criteria for PNSTs. In human medicine, the expression of S-100 protein is used to differentiate between spindle cell tumours of neural and non-neural origins [27]. In veterinary medicine, immunohistochemical detection of S-100 and vimentin has been able to distinguish conclusively between subsets of such spindle cell tumours [28].

This report describes the histologic and immunohistochemical diagnosis of a neurofibrosarcoma in the ulnar of a dog.

## Case presentation

An 8-year-old, 9 kg, female, mixed-breed dog referred to the Small Animal Clinic of Tehran University. Clinical examination revealed a rapidly growing, nodular, subcutaneous mass, 7×4 cm in diameter, invading and strongly adhering to the underlying tissue. The mass was located on the upper right side of the ulnar region. The dog had anorexia, general weakness and inability to stand. Ultrasonography revealed a subcutaneous mass with a central depth of 5.4 cm. ventrally, the margins of the lesion appeared to be well defined and the abdominal organs were not visibly affected.

The blood cell count was undertaken manually and calcium and phosphorus concentration were measured by commercial kits (Pars Azmoon, Alborz, Iran) using a semi-automatic analyzer (EMP 168 Vet Biochemical analyzer; Shenzhen Emperor Electronic technology Co. Ltd, Shenzhen, China). Haematological and biochemical profiles (including blood cell count and serum calcium and phosphorus concentrations) were within normal ranges.

For partial excisional biopsy, an intravenous combination of diazepam (0.27 mg/kg) (Tamin, Tehran, Iran) and ketamine hydrochloride (5.50 mg/kg) (Alfasan, Woerden, the Netherlands) were used for induction and maintenance of anesthesia and the dog received normal saline solution 0.9% intravenously, to a total of 0.5 L (12 mL/kg/h) (Samen, Mashhad, Iran). Atropine sulphate (0.03 mg/kg) (Tamin, Tehran, Iran) was given subcutaneously as pre-medication. The mass was removed surgically and processed routinely. The sample was fixed in formalin and embedded in paraffin for sectioning. The sections were stained with haematoxylin and eosin. For further study, paraffin sections were stained immunohistochemically with S-100, vimentine markers (Abcam Co., Cambridge, USA).

For immunohistochemistry, sections from tumor were mounted on adhesive-coated slides (Superfrost Plus, Menzel-Glaser, Braunschwaig, Germany), processed through xylene, and rehydrated in ethanol. Antigen retrieval was by boiling in a microwave oven (700 W) twice for 5 minutes in Tris–EDTA buffer—1.21 g Tris base (A 1379, Applichem, Darmstadt, Germany) and 0.372 g EDTA (8418, Merck, Darmstadt, Germany)—in 1 liter of distilled water and pH 9. Endogenous peroxidase was blocked with 0.6% (v/v) H_2_O_2_ in Tris-buffered saline (TBS; pH 7.6) for 15 minutes at 20°C before the antibodies used included those for vimentin (prediluted, monoclonal: V9), S-100 protein (1:4,800, polyclonal rabbit anti-S-100).

## Histopathology

Histopathologically, neurofibrosarcoma tumour cells were not circumscribed by connective tissue and neoplastic cells often exhibited an aggressive behavior, high cellularity, cellular pleomorphism, and various morphologic patterns. Atypical mononuclear or multinucleated cells were consistently observed. More than three mitotic figures per high-power field (400×) were found in this case (Figure 1B and 1C). Necrotic foci accompanied by pseudopalisading (Figure 2A) and infiltrates of various numbers of lymphocytes, plasma cells, and macrophages were common.

**Figure 1:** **A: The cells are in disorganized fascicles with pleomorhism, nuclear atypia and neoplastic spindle cells with wavy eosinophilic cytoplasmic processes.** (H & E; bar 20 μm; ×400). **B**: the neoplastic cells form dense bundles separated by scanty collagenous stroma. Notice bland nuclei lacking atypia. (H & E; bar 30 μm; × 400) **C**: Upon histopathological examination of the ulnar mass, neurofibroma with a mixture of round and spindle shaped cells, mitotic figures, infiltrates of various numbers of lymphocytes and hypercellularity arrangement was diagnosed. (H & E; bar 25 μm; × 400).

**Figure 2:** **A: Necrotic focus is accompanied by nuclear pseudopalisading in MPNST, 2B: Neoplastic cells with cytoplasm and round nuclei are arranged in a cordlike pattern, 2C: The neoplastic cells show diffuse expression of S-100.** IHC, **2D**: The neoplastic cells show strong expression of vimentin. IHC **2E**: A number of neoplastic cells show a marked cytoplasmic and nuclear immunoreaction for S-100 protein **2F**: Fusiform or spindle-shaped neoplasmic cells are arranged in interdacing fascicles.

In some areas, neurofibrosarcoma was composed mainly of a homogeneous population of round cells (Figure 1C). These round cells were arranged in sheets or cords with a meshwork of intratumoral nerve fibers. The nuclei were round or oval (Figure 1A and 2B). Furthermore, in some areas, the spindle cells had long wavy nuclei with tapered ends. Some had oval, round, short spindle nuclei, or had nuclear pseudo-inclusions (Figure 3A, 3B and Figure 1A, 1C).

**Figure 3:** Immunohistochemical staining with, vimentin (A) and S-100 (B and C) are positive cells; the neoplastic cells in parts of the neurofibroma express S-100 and vimentin strongly.

However, in some regions of the tumor tissue, fusiform or spindle cells arranged in densely or loosely sweeping fascicles, interlacing whorls, or storiform patterns together with wavy cytoplasm, nuclear palisades were predominant (Figure 2F). In addition, the neoplastic cells within the blood vessels were observed as well.

Immunohistochemical features of the spindle-shaped neoplastic cells were predominantly positive for S-100 and vimentin (Figure 3A, 3B and 3C) and the cytoplasm and/ or nucleus of the neoplastic cells were diffusely labeled for expression of vimentin (Figure 2D), S-100 (Figure 2C and 2E).

## Discussion

PNSTs have also been reported in cats, dogs, cattle, rats, and horses [3,29,30]. In human, these tumours have been subclassified as neurinomas, neurilemmomas, schwannoma, neurofibromas, neurofibrosarcomas, and malignant peripheral nerve sheath tumors (MPNSTs), based on their presumed cell(s) of origin. In the dog, 2 groups of tumors have been referred to as PNSTs, 1 occurring in the cranial and spinal nerves and 1 occurring in the skin and subcutaneous [31].

Many of the first group are consistent with MPNSTs and have metastatic potential [3]. Those occurring in the skin and subcutaneous of dogs are usually of uncertain histogenesis and are referred to by some as hemangiopericytoma [32]. Palisading, as seen in classic PNSTs, is usually absent [31].

The histological differentiation between malignant and benign PNST can be difficult because both may show undefined edges and some degree of cellular pleomorphism [33]. It has been suggested that malignant PNST in dog have aggressive behavior to intratumoral tissue, extensive necrotic areas and cellular pleomorphism [34-36]. All of these characteristics were observed in this case; however, the presence of neoplastic cells within the blood vessels was observed that determined the classification of malignancy. A high level of mitosis is also indicative of a malignant PNST [34,36]. In present study, the malignant histological appearance of the lesion (mitotic index, cellular pleomorphism or necrosis) occurred in conjunction with infiltrative growth.

In dogs and humans, divergent differentiation is usually associated with a poor prognosis [21,37]. The S100 protein is the primary marker in the diagnosis of MPNST (malignant schwannoma*,* neurofibrosarcoma*,* and neurogenic sarcoma) and may be used as a single diagnostic tool [38,39] or in combination with other markers such as vimentin [40,41]. The neoplastic cells in this study showed positivity for S100 and vimentin immunolabeling.

In this study, based on their morphologic features diagnostic for human neurofibrosarcoma, i.e., growth pattern and microscopic features (such as areas of high cellularity, cellular pleomorphism, various morphologic patterns, high mitotic index and high number of undifferentiated neoplastic cells), together with the presence of intratumoral nerve fibers and the restriction of the S100 and vimentin immunostaining to a subpopulation of the neoplastic cells, the tumour was diagnosed as neurofibrosarcoma. But the cause of MPNST in domestic animals has not yet been determined. Due to its anatomical location and difficulties encountered in complete surgical removal. Canine MPNST often recurs after surgery and the prognosis is generally poor [42]. In addition, the prognosis of human patients with primary MPNST is poor and removal is often followed by recurrence, metastasis and death [43-45]. No definitive evidence of distant organ metastasis was found in this case.

Neurofibrosarcoma in this report had marked morphologic variation. The round cell type found in this case was morphologically similar to the primitive neuroectodermal tumour described as the small round-cell type in human MPNST [46] or one of the malignant schwannomas [47], suggesting that the presence of round cells implies a differentiation toward immature neural cells.

Immunohistochemical expression of S100 protein and vimentin by the neoplastic cells prompted consideration of peripheral nerve sheath tumour in the differential diagnosis. Various immunohistochemical markers have been used to define MPNST. S-100 is commonly expressed in normal nervous tissue and in most MPNST [48], but also in most rhabdomyosarcomas and neurofibrosarcoma [49]. The present case was positive for expression of vimentin and S-100.

On the basis of gross morphology, histopathological and immunohistochemical features, the final tumour in this study, a diagnosis of neurofibrosarcoma was made. For understanding of these complex neoplasms and the development of the effective differential diagnosis, further investigation will be needed into the clinical features and the basic science.

## Conclusion

This study described histopathology and immunohistochemical features of canine subcutaneous neurofibrosarcoma of the ulnar region. The histological features of these tumours would suggest that most should be classified as high-grade MPNST. A subcutaneous MPNST may be diagnosed on the basis of observing the histopathological pattern described in present study. In addition, S-100 and vimentin immunohistochemical expression may be used to help confirm the diagnosis of neurofibrosarcoma. Finally, the use of immunohistochemistry may be helpful in distinguishing this type of neoplasm from other malignancies with similar morphology. The incidence of neurofibrosarcoma in animals is unknown; we hope this will become clearer. To our knowledge, this is the first report of ulnar MPNST in a dog, suggesting that this tumour should be included as a differential diagnosis for ulnar spindle cell tumours.

## Competing interests

The authors declare that they have no competing interests.

## Authors’ contributions

AT and FK participated in the histopathological evaluation, performed the literature review, acquired photomicrographs and drafted the manuscript and gave the final histopathological diagnosis. JJperformed sequencing alignment and manuscript writing. EH and AB carried out the immunohistochemical stains evaluation. MAH and MMM edited the manuscript and made required changes. All authors have read and approved the final manuscript.
